RETRACTED

# Effect of IMB Model Combined with Spousal Support Breastfeeding Intervention on PBSES Score and Breastfeeding Rate of Primipara with Chronic Hepatitis B Virus Infection

**DOI:** 10.1155/2022/9661408

**Published:** 2022-09-15

**Authors:** Shaoping Chen, Linxian Li, Qianwen Sun, Shulan Chen, Jing Cheng, Siqi Xiong

**Affiliations:** ^1^Obstetrics Department, National Clinical Research Center for Infectious Disease, Shenzhen Third People's Hospital, Shenzhen, Guangdong 518112, China; ^2^Obstetrics Department, The Second Affiliated Hospital of Southern University of Science and Technology, Shenzhen, Guangdong 518112, China

## Abstract

**Objective:**

To analyze the effects of the info-motivation-behavior skills (IMB) model combined with spousal support breastfeeding intervention on breastfeeding Self-Efficacy Scale (PBSES) scores and breastfeeding rate of primiparas with chronic hepatitis B virus (HBV) infection.

**Methods:**

Seventy-four first-term pregnant women and 74 of their spouses were selected as the traditional control group by the convenience sampling method from July to September 2021 in obstetrics department of Shenzhen Third People's Hospital. 74 pregnant women with their first child and 74 spouses who had their first child checked during October to December 2021 were classified as the IMB model group. The traditional control group was applied with conventional intervention management mode, and the IMB model group was applied with intervention management mode based on IMB theory on the basis of the traditional control group. The self-efficacy scores of breastfeeding before and after intervention during pregnancy and during hospitalization were compared between the two groups, and the self-efficacy scores of paternal support for breastfeeding were compared. The exclusive breastfeeding rate of infants within 6 months and the maternal breastfeeding knowledge level of the two groups were compared, and the correlation between maternal breastfeeding self-efficacy score and feeding knowledge level was analyzed.

**Results:**

After pregnancy intervention, PBSES and FBSES-SF scores were significantly increased in both groups, and scores of scales in the IMB model group increased significantly than the traditional control group (all *P* < 0.05). The BSES-SF and FBSES-SF scores of the IMB model group increased significantly than the traditional control group at 3 days after delivery and at discharge (*P* < 0.05), and the scores of each scale at discharge in both groups increased significantly than those at 3 days after delivery (*P* < 0.05). The rate of exclusive breastfeeding in the IMB model group was 94.59% (70/74), and that in the traditional control group was 78.38% (58/74). There was a significant difference (*χ*2 = 8.325, *P* = 0.004). At discharge, the score of maternal breastfeeding knowledge increased significantly in both groups, and the score of the IMB model group increased significantly than that of the traditional control group (all *P* < 0.05). Pearson correlation coefficient was used to analyze the correlation between PBSES score, FBSES-SF score, and maternal feeding knowledge level, which showed positive correlation (all *P* < 0.05).

RETRACTED

**Conclusion:**

The self-efficacy of prenatal breastfeeding in pregnant women with HBV is low, and the application of the IMB model combined with the intervention mode of spy-supported breastfeeding has positive effects on the improvement of maternal breastfeeding efficiency, breastfeeding health knowledge level, and postpartum breastfeeding rate, which is worthy of clinical promotion and application.

## 1. Introduction

Breast milk is an essential food for infants in the first six months after birth. In addition to a variety of nutrients, breast milk also has a variety of bioactive substances, which have positive significance in enhancing immunity and promoting intellectual development of infants [1, 2]. Breastfeeding reduces the risk of respiratory diseases and diarrhea in infants and reduces infant mortality. Breastfeeding can also promote postpartum recovery, improve parent-child bond, and reduce the risk of diabetes, breast cancer, and ovarian cancer in mothers [3]. The World Health Organization and UNICEF recommend early initiation of breastfeeding and exclusive breastfeeding of infants under 6 months for optimal growth [4, 5]. In 2019, the National Nutrition Survey and special investigation on breastfeeding found that the exclusive breastfeeding rate of 6-month-old infants in China was about 30% [6], which is far from the national nutrition plan's target of 50% by 2020. Due to viral load, family opposition, and fear of mother-to-child transmission, the actual postpartum exclusive breastfeeding rate of pregnant women infected with hepatitis B virus (HBV) in China is not high [7]. Promoting breastfeeding is an important basic work for ensuring maternal and child health and promoting the construction of a healthy China. The info-motivation-behavior skill (IMB) model is a kind of health education model emerging in recent years. The application of the IMB model can help education objects better accept knowledge and master skills. The application of the IMB model can help learners stimulate subjective initiative and enthusiasm, and the theoretical model has been recognized in the application of breastfeeding management in foreign countries. The theoretical model has been recognized in the management of breastfeeding in foreign countries. Based on this, based on the recent domestic and foreign research progress in effectively promoting breastfeeding behavior, this study used mature and feasible “IBM model” as a health education behavioral intervention method for pregnant women and their spouses during the pregnancy and perinatal period, combined with two strategies of breastfeeding self-efficacy and father's support for breastfeeding. Main information intervention of maternal pregnancy and motivated interviews, encourage the spouse support and help first-time mothers build confidence, keep the exclusive breastfeeding behavior and behavioral interventions to assist the breastfeeding operating skills as soon as possible, and observe the intervention model to improve breastfeeding rates and promote maternal and child health, such as effectiveness, is presently as follows the results of the study report.

RETRACTED

The basic structure of this paper is as follows: The standard focus-IMB model combined with spousal support for breastfeeding intervention program is described in detail in Section 2.2.2 of this paper. The clinical effects and other relevant research data of the intervention program are presented in Part 2. The conclusions of this study based on IMB model and related research results of spousal-supported breastfeeding intervention program are described in detail in the third part.

## 2. Data and Methods

### 2.1. General Information

Seventy-four first-term pregnant women and 74 of their spouses were selected as the traditional control group by the convenience sampling method from July to September 2021 in obstetrics department of Shenzhen Third People's Hospital. 74 pregnant women with their first child and 74 spouses who had their first child checked during October to December 2021 were classified as the IMB model group. In the traditional control group, mothers ranged in age from 21 to 35 years old, with an average of (27.19 ± 3.46) years old. There were 42 cases with college degree or above, 22 cases with secondary school/high school degree, and 10 cases with junior high school degree. The age of fathers ranged from 23 to 37 years old, with an average of (28.23 ± 4.34) years old. There were 45 cases with college education or above, 20 cases with secondary school/high school education, and 9 cases with junior high school education. In the IMB model group, the maternal age ranged from 22 to 36 years old, with an average of (27.64 ± 3.75) years old. 40 cases had college degree or above, 25 cases had technical secondary school/high school degree, and 9 cases had junior high school degree. The age of fathers ranged from 21 to 37 years old, with an average of (28.82 ± 4.94) years old. 44 cases had college education or above, 22 cases had secondary school/high school education, and 8 cases had junior high school education. There was no significant difference in age, education level, and other general information of puerpera and spouse (*P* > 0.05).

RETRACTED

Inclusion criteria were as follows: (1) both husband and wife are over 18 years old and have received primary school education or above; (2) the diagnostic criteria for pregnant women with chronic HBV infection were based on clinical guidelines for prevention of mother-to-child transmission of hepatitis B virus (2020) [8]: HBsAg positive duration > 6 months and normal liver function, quantitative detection of HBV DNA before delivery: ≤2 × 10^5^kIU/L (IU/mL), and no need to take HBV antiviral drugs after delivery; (3) all of them were born naturally in a single child, willing to breastfeed after delivery, and signed written informed consent; (4) are for the term birth, birth 1, and 5 min Apgar scoring for 8 ~ 10 points (after birth, respectively, from the heart rate, respiration, skin color, muscle tension, throat five aspects reflected in Alzheimer's rating normal newborns), and newborn babies are born within 12 hours after inoculation of hepatitis b immune globulin 10 mu g 100 U and recombinant hepatitis b vaccine.

Exclusion criteria were as follows: (1) pregnant women who are taking therapeutic drugs (e.g., antivirals) whose safety for the infant is uncertain; (2) pregnancy complicated with hepatitis C, syphilis, AIDS, and other infectious diseases; (3) those who still choose to give up breastfeeding after medical education and guidance; (4) cognitive impairment and mental illness; (5) and do not deliver in this hospital. Neonates were transferred to the neonatology department after discharge.

### 2.2. Intervention Methods

#### 2.2.1. Traditional Control Group Intervention Method

Prenatal was as follows: paper health education pamphlets and 12 online school courses for pregnant women during pregnancy: hepatitis B disease knowledge and maternal and infant prevention measures are routinely distributed after the establishment of the file and delivery examination. Breastfeeding principle and feeding benefits measure to maintain breast milk secretion. The breastfeeding position connects with the infant and causes solving skills of common breastfeeding problems and measures for breast milk storage, chasing, and carrying; observation and nursing of neonatal jaundice and breast feeding jaundice; newborn bath, umbilical cord, and skin care; diet, rest, exercise, and emotional regulation during breastfeeding. There are specific spousal support measures during breastfeeding, and there is physiological phenomena of newborn. The newborns were followed up after 0 ~ 6 months of vaccination and hepatitis B vaccine vaccination. Each lesson lasts 5 ~ 10 minutes. It can be viewed repeatedly. Video homemade or purchase was push through WeChat.

RETRACTED

Postpartum was as follows: nurse in postpartum mission of the benefits of breastfeeding and the disadvantages of artificial feeding and manual by oral education, health education, and demonstration in the form of guidance and correct nursing instruction emphasizes the newborns with nipple, right to avoid bleeding, cracked nipples when mothers found cracked nipple, can stop breastfeeding, and return after being improved. Observe the newborn mouth closely for any discomfort such as ulceration, ulcer, herpes, and bleeding.

Discharge guidance was as follows: clinical medical staff inform parturients and their families of the importance of breastfeeding and guide parturients to massage the breast and deal with the phenomenon of milk rise. The medical staff should let the puerpera pay attention to the situation that the baby is prone to bite the mother's nipple in the teething stage and guide the puerpera to pay attention to and maintain the correct feeding posture in the process of breastfeeding. Infants should have their own independent tableware, and their families need to boil, disinfect, and dry their tableware before using them.

#### 2.2.2. Intervention Methods in IMB Model Group

On the basis of the traditional control group, breastfeeding intervention program based on IMB theory and spousal-supported breastfeeding dual theory was implemented. The specific interventions were as follows: (1) information intervention: 12 online school courses for pregnant women during pregnancy, the contents of which were the same as those of the control group, and (2) motivational intervention: motivational interviews were used to conduct 1 to 2 interventions for pregnant women and their spouses, in order to mobilize the motivation of pregnant women and their spouses to support, and interviews were conducted around 5 periods of behavior change, including pregnant women 16 to 20 weeks of pregnancy (no intention period), 24 to 28 weeks of pregnancy (intention period), 30 to 34 weeks of pregnancy (preparation period), 36 to 38 weeks of pregnancy (change period), the day of admission (maintenance period), and 15 to 30 minutes per time. Interviews were conducted with pregnant women's spouses as family units, centering on the most concerned information such as hepatitis B disease knowledge, mother-to-child prevention program, and benefits of breastfeeding. According to the first measurement scale, targeted solutions and discussions were carried out to realize the importance of exclusive breastfeeding: targeted solution and discussion for the second measurement scale, correct traditional misconceptions (such as adding milk powder to sleep better and grow faster), and build confidence in exclusive breastfeeding. Individualized guidance for the mastery of common breastfeeding problem solving skills. Evaluating and revising exclusive breastfeeding programs to ensure their viability. According to the preliminary investigation and interview results, targeted and individual intervention was conducted after on-site evaluation of postpartum maternal and infant situation. Encourage spouses to support and assist new mothers, e.g., through verbal encouragement, action, and emotional support, to build confidence and maintain exclusive breastfeeding behavior. (3) Behavioral intervention was as follows: after the puerpera returned to the ward after delivery, the nurse in the management bed explained the situation of the implementation of neonatal hepatitis B immunoglobulin injection, hepatitis B vaccine vaccination, the benefits and effects of hepatitis B mother-to-child blocking, and concerns about contact with breastfeeding; When the puerpera is willing to cooperate within 2 hours after returning to the ward after delivery, the first bedside guidance will be given with the spouse observing and learning. Nursing bed nurses demonstrate breastfeeding operation, guide maternal breastfeeding posture, help newborn in the postpartum ward for the first time skin contact with the nipple and nipple connection, help newborn to correctly contain most of the nipple areola, and at the same time, guide puerperians and their spouses to watch the “breastfeeding” course in online school courses for pregnant women, so as to help them master the operation skills of breastfeeding as soon as possible. On the first day after delivery, the puerpera and her spouse were guided to breastfeeding operation. The nursing nurse watched and provided correct guidance continuously and encouraged her to repeat training. The responsible leader or head nurse conducted on-site assessment every day to help puerpera and her spouse master and consolidate breastfeeding operation. Between the third day after delivery and discharge from hospital, there was a nursing staff to guide primipara and spouses to watch online in pregnant women school curriculum “newborn care” “neonatal physiological phenomenon” in combination with breastfeeding practice, aiming at the existence of breastfeeding in the question, such as milk deficiencies, problems such as sore nipples, rose milk, and tube bed, answer them one by one and correct guidance, to help mothers and spouse build confidence, and keep the exclusive breastfeeding behavior. Within 2 weeks after the puerpera was discharged from hospital, the puerpera and their spouse were, respectively, visited by telephone. The contents of the visit were about breastfeeding, the questions raised by the puerpera and their spouse were answered in time, and the puerpera and their spouse were encouraged to adhere to exclusive breastfeeding. In the return visit of the puerpera, the participation of the spouse was asked, and the return visit of the spouse was affirmed and encouraged. 6 to 8 weeks after delivery, inform the puerpera to make an appointment with the breastfeeding clinic in time, evaluate the breastfeeding process on site, and solve the problem accordingly.

RETRACTED

### 2.3. Observation Indicators

1. The scores of breastfeeding self-efficacy and paternal support for breastfeeding self-efficacy were compared between the two groups before and after intervention during pregnancy
2. Maternal breastfeeding self-efficacy scores and paternal breastfeeding self-efficacy scores were compared between the two groups from the 3rd day after delivery in hospital to before discharge
3. The rate of exclusive breastfeeding in 6 months was compared between the two groups
4. The knowledge level of maternal breastfeeding was compared between the two groups
5. To analyze the correlation between maternal breastfeeding self-efficacy score and feeding knowledge level
6. Comparing the mother-to-child transmission rate of HBV-DNA

### 2.4. Evaluation Criteria

Paper questionnaires were used to investigate all subjects and their spouses. The spouse would fill out a Father Support Breastfeeding Self-Efficacy Scale-Short Form (FBSES-SF), which was developed by Dennis [9]. A total of 14 items were used to measure fathers' confidence in supporting breastfeeding. The Likert 5-level scoring method was used for each item, with a total score of 14-70 (“1= not at all confident” to “5= very confident”). The higher the score, the stronger the fathers' self-efficacy in supporting breastfeeding.

Prenatal Breastfeeding Self-efficacy Scale (PBSES) and Breastfeeding self-efficacy Scale (PPI) are completed by first-time mothers' scale, and BSES-SF is used to measure maternal confidence in self-adherence to breastfeeding behavior at different stages. PBSES scale is Likert grade 5 (“1= not at all confident” to “5= very confident”), with a total score of 20-100, and the higher the score, the better the maternal self-efficacy of prenatal breastfeeding [10]. The BSES-SF scoring scale also adopts the Likert grade 5 scoring method, with a total score of 14-70. The higher the score is, the stronger the maternal self-efficacy of breastfeeding is, and the more likely it is to tend to exclusive breastfeeding [11]. All subjects were given various questionnaires before the first pregnancy intervention, after the pregnancy intervention, on the day of admission, and on the day of discharge. All questionnaires were effectively collected. The questionnaire on breastfeeding knowledge was designed by Zhao [12], a scholar, after referring to domestic and foreign literatures, to measure the knowledge level of breastfeeding of primiparas. The 17-item questionnaire asked about the benefits and skills of breastfeeding. One point is given for each item answered correctly, and the total score ranges from 0 to 17. The higher the score, the more knowledge primiparas have about breastfeeding. Exclusive breastfeeding rate within 6 months after delivery (number of newborns exclusively breastfed within 6 months after delivery/total number of newborns included in this study × 100%) was calculated.

RETRACTED

### 2.5. Statistical Treatment

The collected data were processed by SPSS 26.0 software, and the unit of measurement data conforming to normal distribution was mean ± standard deviation (^−^*x* ± *s*). *t*-test was performed for data differences within and between groups. Counting data were expressed by (*n*, %), and data differences between groups were analyzed by *x*^2^ test. Pearson correlation coefficient was used to analyze breastfeeding self-efficacy score and feeding knowledge level. *P* < 0.05 indicated significant differences in data results, with statistical significance.

The greater the absolute value of the correlation coefficient, the stronger the correlation: the closer the correlation coefficient is to 1 or -1, the stronger the correlation; the closer the correlation coefficient is to 0, the weaker the correlation.

## 3. The Results

### 3.1. Comparison of PBSES and FBSES-SF Scores before and after Intervention during Pregnancy

Before pregnancy intervention, there were no significant differences in PBSES and FBSES-SF scores (all *P* > 0.05), but after pregnancy intervention, the PBSES and FBSES-SF scores were significantly increased, and the scales scores of the IMB model group increased significantly than the traditional control group (all *P* < 0.05), as shown in Table 1.

### 3.2. The Maternal BSES-SF and Father FBSES-SF Scores Were Compared from the Third Day after Delivery in Hospital to the Time of Discharge

The scores of BSES-SF and FBSES-SF in the IMB model group were significantly higher 3 days after delivery and at discharge than those in the traditional control group (*P* < 0.05), and the scores of each scale at discharge in both groups increased significantly than those at 3 days after delivery (*P* < 0.05), as shown in Table 2.

RETRACTED

### 3.3. The Rate of Exclusive Breastfeeding within 6 Months Was Compared

The rate of exclusive breastfeeding in the IMB model group was 94.59% (70/74), and that in the traditional control group was 78.38% (58/74). There was a significant difference (*χ*^2^ = 8.325, *P* = 0.004).

### 3.4. The Knowledge Level of Maternal Breastfeeding Was Compared

There was no significant statistical difference in the scores of maternal breastfeeding knowledge at admission (*P* > 0.05), but the scores of maternal breastfeeding knowledge at discharge were significantly increased, and the scores of the IMB model group increased significantly than the traditional control group (both *P* < 0.05), as shown in Table 3.

### 3.5. Analyze the Correlation between Maternal Breastfeeding Self-Efficacy Score and Feeding Knowledge Level

Pearson correlation coefficient was used to analyze the correlation between PBSES score, FBSES-SF score, and maternal feeding knowledge level, which showed positive correlation (all *P* < 0.05), attached Figures 1 and 2.

## 4. Discussion

IMB model is a scientific, personalized, and sustainable health education behavior mode, which is suitable for carrying out effective breastfeeding behavior intervention during pregnancy as a theoretical guidance and behavior intervention mode. The theory holds that information factor, motivation factor, and behavior skill factor are three core factors of behavior establishment. Information factor refers to specific health knowledge, motivational factor includes personal motivation (individual attitude towards health behavior) and social motivation (social support), and behavioral skill factor mainly refers to objective skills for establishing behaviors [13]. The advantage of the IMB model is that it considers the influence of social psychological factors on behaviors and believes that individual's attitude, perceived social support, and self-efficacy play a key role in health behavior prevention intervention. It integrates information, psychological, and social factors together to establish healthy behaviors from an overall perspective. At the present stage, it has been widely used in the health education of patients with clinical aids, hypertension, and surgical surgery and achieved good results [14].

Breastfeeding is a fragile and variable behavior that is susceptible to a variety of factors. Under the influence of China's traditional concept, breastfeeding is considered to be a natural process led by the puerpera, and the traditional concept of “men take care of the outside and women take care of the inside” leads to the low level of support for breastfeeding by the spouse. Breastfeeding is a highly recommended way of parenting in clinical practice. At the same time, breastfeeding is conducive to improving postpartum uterine contractions, promoting maternal physical recovery, and promoting maternal and infant feelings. However, due to the maternal cesarean section postoperative pain, coupled with the lack of understanding of the benefits of exclusive breastfeeding, it is not high enthusiasm for exclusive breastfeeding. Education during pregnancy can promote the rate of postpartum exclusive breastfeeding [15]. In addition, previous studies show that while the father cannot directly provide milk, but positive attitude, and practice in the whole process of breastfeeding support and emotional encouragement will directly affect the maternal breastfeeding self-efficacy and the higher maternal breastfeeding self-efficacy, tending to the greater the chance of exclusive breastfeeding [16]. In this study, after intervention during pregnancy, PBSES and FBSES-SF scores were increased significantly than before intervention, and the scores of the subjects receiving the IMB model combined with spousal support intervention program were significantly higher than those of the traditional control group (all *P* < 0.05). Comparison of bSES-SF and FBSES-SF scores between the two groups showed a significant increase during hospitalization, but the scores of subjects receiving the IMB model combined with spouse support intervention program increased significantly than those of the traditional control group (all *P* < 0.05), and the knowledge level of maternal and infant feeding was also significantly higher. It is suggested that IMB model-based breastfeeding health education for primiparas and their spouses is more helpful to improve the breastfeeding self-efficacy of primiparas, which is basically consistent with previous research results. It may be related to the emphasis on spouse intervention. Breastfeeding is a fragile and variable behavior, many women feel weak after childbirth due to fatigue, weakness, wound pain, and other physiological and psychological reasons, and mood is not good; in addition, in the long-term breastfeeding process that may appear less milk, baby crying, nipple pain, and other factors are affecting maternal adherence to breastfeeding. In this process, spousal support can play a huge role. In this study, the intervention group had a good impact on breastfeeding by emphasizing the role of spousal support. Although the spouse cannot provide breast milk directly, the positive attitude, practical support, and emotional encouragement in the whole process of breastfeeding will directly affect the maternal breastfeeding self-efficacy, and the higher the maternal breastfeeding self-efficacy, the greater the likelihood of exclusive breastfeeding. As the first caregiver, the spouse has the most time to accompany the parturient, and its positive attitude, emotional encouragement, and action support will directly affect the parturient's mentality and breastfeeding behavior. Maternal lactation is regulated by hormone level, which is closely related to mental and psychological state. The attention and emotional love of the spouse can help the maternal to adjust negative postpartum mentality as soon as possible, which is conducive to lactation. In addition, the improvement of maternal breastfeeding self-efficacy also benefits from online schools, and pregnant women online school curriculum is especially suitable for beginners learning and can repeat playback, convenient primipara, and spouses of learning, to help new parents' idea which is consistent and common to solve the difficulties in the process of breastfeeding, to establish the confidence of exclusive breastfeeding. Thus, it can improve the self-efficacy of breastfeeding for primiparas [17, 18]. In addition, this study is aimed at maternal breastfeeding self-efficacy scores and mother's milk which is correlation analysis knowledge level and shows a significant positive correlation (*P* < 0.05), suggesting in clinical nurse in a planned way, step by step, targeted to the implementation of the guidance of breastfeeding, to ensure that the path in the table all the projects are implemented and to promote the maternal knowledge and skills of breastfeeding in a comprehensive system. Adequate knowledge and good feeding skills of pregnant women will lay a good foundation for their persistence and success in breastfeeding and improvement of self-feeding efficiency.

RETRACTED

It is important to note that because of HBV infection in pregnant women for breastfeeding inherent cannot breastfeed and increase the risk of mother-to-child transmission of entrenched idea influence, they need to strengthen health education and advocated the spouse during pregnancy, postpartum main family-centered care family members should participate in, and second liver disease knowledge and breastfeeding education project will be conducive to improve the level of exclusive breastfeeding family support, help HBV-infected pregnant women and their families to break the traditional inherent concepts of breastfeeding, and eliminate the inherent ideas of pregnant women and their families with successful cases of breastfeeding [19, 20]. The results of this study showed that the maternal breastfeeding rate of the IMB model group increased significantly than that of the traditional control group (*P* < 0.05). The lack of breastfeeding knowledge is the main reason for the decline in the rate of postpartum exclusive breastfeeding. The results of this study suggest that HBV breastfeeding knowledge level is an important factor affecting prenatal breastfeeding self-efficacy of pregnant women with HBV. The higher the level of breastfeeding knowledge, the greater the confidence in breastfeeding and the higher the self-efficacy of breastfeeding. At the same time, standard and good breastfeeding skills are the premise to ensure the safety of breastfeeding, and it is very important to master the characteristics of HBV feeding, which is also an important mechanism to improve the safety of breastfeeding. For example, in the process of feeding, when the puerpera has adverse symptoms such as nipple rupture and bleeding, or the newborn has oral ulcer, oral herpes, diarrhea, and other symptoms, the puerpera should suspend the breastfeeding of the newborn, to avoid the HBV in the milk directly through the damaged mucosa into the baby's blood [21]. Puerpera and babies should often trim their nails and keep them clean, so as not to scratch the skin and mucous membrane and reduce the risk of infection. Baby tableware should be used alone, boiled before use disinfection, and dry storage. Medical staff should strengthen prenatal propaganda and education of HBV pregnant women with breastfeeding knowledge through classes for pregnant women and other ways to help them master breastfeeding skills and can also provide one-to-one guidance through breastfeeding consultation clinics to improve the breastfeeding rate and ensure the safety of breastfeeding [22]. Some scholars [23] conducted a qualitative interview study on pregnant women carrying HBV and found that most pregnant women did not know about the transmission route of HBV, mother-to-child blocking measures, and HBV testing of their children. It indicates that there is insufficient knowledge education for this special group, which leads to their cognitive deviation of breastfeeding and reduces the self-efficacy of breastfeeding. Therefore, it is very important for pregnant women carrying HBV to obtain scientific knowledge of HBV transmission and mother-to-child blocking through professional education and guidance of medical staff, so as to remove their concerns about breastfeeding and accept the new concept of breastfeeding. The form of propaganda and education can provide various forms of support for pregnant women, such as schools, prepregnancy check-ups, WeChat public accounts, online classes, and pamphlets, as well as WeChat, QQ, telephone, and door-to-door services, so as to timely solve their problems and improve their prenatal breastfeeding self-efficacy. Collaboration between relevant disciplines should also be strengthened, and consensus should be reached among members to avoid conflicting views, which may lead to conflicting knowledge for pregnant women and their families [24].

RETRACTED

## 5. Conclusion

In conclusion, the safety of breastfeeding in pregnant women carrying HBV is getting higher and higher. In view of the advantages of breastfeeding, they should be encouraged to choose breastfeeding as much as possible. The self-efficacy of prenatal breastfeeding in pregnant women with HBV is low, and the application of the IMB model combined with the intervention mode of spy-supported breastfeeding has positive effects on the improvement of maternal breastfeeding efficiency, breastfeeding health knowledge level, and postpartum breastfeeding rate, which is worthy of clinical promotion and application.

## Figures and Tables

**Figure 1:** Correlation between PBSES score and breastfeeding knowledge score.

**Figure 2:** Correlation between BSES-SF score and breastfeeding knowledge score.

**Table 1:** Comparison of PBSES and FBSES-SF scores between the two groups before and after intervention during pregnancy.

Group	PBSES scores		FBSES-SF scores	
	Before intervention	After intervention	Before intervention	After intervention
IMB model group (*n* = 74)	28.76 ± 3.23	74.17 ± 8.43^∗^	27.11 ± 2.46	57.46 ± 6.47^∗^
Traditional control group (*n* = 74)	29.38 ± 3.45	51.33 ± 6.35^∗^	26.72 ± 2.23	35.96 ± 4.52^∗^
*t*	-1.129	18.616	1.010	23.434
*P*	0.261	<0.001	0.314	<0.001

Note: ^∗^ represents comparison with before intervention, *P* < 0.05.

**Table 2:** Comparison of maternal BSES-SF and father FBSES-SF scores from the 3rd day after delivery to before discharge to discharge.

Group	BSES-SF score		FBSES-SF score	
	3 days after delivery	When out of the hospital	3 days after delivery	When out of the hospital
IMB model group (*n* = 74)	52.15 ± 3.52	59.49 ± 7.56^∗^	47.85 ± 2.56	58.37 ± 8.04^∗^
Traditional control group (*n* = 74)	47.58 ± 3.59	51.14 ± 5.53^∗^	43.33 ± 2.74	47.16 ± 6.58^∗^
*t*	11.241	8.587	10.369	9.282
*P*	<0.001	<0.001	<0.001	<0.001

Note: ^∗^ represents *P* < 0.05 compared with 3 days after delivery.

**Table 3:** Comparison of maternal breastfeeding knowledge score.

Group	On admission	When out of the hospital
IMB model group (*n* = 74)	9.25 ± 1.06	14.26 ± 1.51^∗^
Traditional control group (*n* = 74)	9.17 ± 0.93	11.68 ± 1.26^∗^
*t*	0.488	11.285
*P*	0.626	<0.001

Note: ^∗^ represents comparison with admission, *P* < 0.05.

RETRACTED

## Data Availability

The dataset used in this paper are available from the corresponding author upon request.
